RETRACTED

# The Effect of Symptom Clusters and Sleep Disorder on Quality of Life among Patients with Chronic Obstructive Pulmonary Disease

**DOI:** 10.1155/2021/1692480

**Published:** 2021-08-31

**Authors:** Guihua Hao, Qiaojing Qiu, Lili Hou, Fen Gu

**Affiliations:** ^1^Nursing Department of Shanghai Ninth People's Hospital, Shanghai JiaoTong University School of Medicine, Shanghai, China; ^2^Emergency Department of the Affiliated People's Hospital of Ningbo University, Zhejiang, China

## Abstract

**Background:**

Symptoms (cough, dyspnea, fatigue, depression, and sleep disorder) in chronic obstructive pulmonary disease (COPD) are related to poor quality of life (QOL). Better understanding of the symptom clusters (SCs) and sleep disorder in COPD patients could help to accelerate the development of symptom-management interventions.

**Objective:**

We aim to explore the effect of sleep disorder and symptom clusters on the QOL in patients with COPD.

**Methods:**

223 patients with stable COPD from November 2019 to November 2020 at the Affiliated People's Hospital of Ningbo University in China were included in this cross-sectional survey. A demographic and clinical characteristics questionnaire, the Revised Memorial Symptom Assessment Scale (RMSAS), the Pittsburgh Sleep Quality Index (PSQI), and the St George Respiratory Questionnaire for COPD (SGRQ-C) were completed by the patients. Exploratory factor analysis was conducted to extract SCs, and logistic regression analysis was performed to analyze the risk factors affecting QOL.

**Results:**

Three clusters were extracted: respiratory functional cluster, emotional cluster, and fatigue-sleep cluster. 70.4% of the participants were poor sleepers. Subgroup analysis showed that COPD patients with poor sleep quality were significantly different in QOL, emotional cluster, and fatigue-sleep cluster compared with patients with normal sleep. In multiple regression, sleep quality and respiratory functional cluster were associated with QOL.

**Conclusion:**

In patients with stable COPD, three symptom clusters were explored. Symptom clusters correlate with clinical features and negatively affect QOL. Appropriate interventions are expected to inform future approaches to symptom management. Future studies are needed to test interventions that may be effective at improving the QOL of COPD patients.

## 1. Introduction

Chronic obstructive pulmonary disease (COPD) is characterized by chronic respiratory symptom, persistent airflow restriction, and decline in lung function [1]. The worldwide prevalence is estimated to be 10% among adult population, increasing significantly in elder population. COPD is currently underestimated due to lack of disease awareness and delayed diagnosis in Asian [2]. A nationally representative sample of Chinese adults was assessed in the China Lung Health Research; among 57,779 participants, the prevalence of COPD was 8.6%, which was about 100 million people, which was a serious public health issue [3]. COPD caused more than 3 million deaths in 2017 and was expected to grow to 4.5 million by 2040, making it the 3rd leading cause of death worldwide [4].

RETRACTED

A wide spectrum of physical and psychological symptom experiences occurs in COPD patients, such as cough, dyspnea, fatigue, depression, and sleep disturbance [5, 6]. Symptom is an important but understudied aspect of COPD. Dyspnea is the main symptom of COPD. Shortness of breath was presented in 64.2% of the COPD patients, which could lead to poor QOL [7]. COPD patients with depression and anxiety have poor QOL [8, 9]. In addition, decline in physical function affects symptoms and QOL in patients with COPD [10, 11]. A good night's sleep is the prerequisite for mental and physical health. However, sleep disorders are common among COPD patients; about 72% of patients had trouble sleeping at least once and 50% had trouble sleeping more than three times a week [12]. Notably, it is increasingly recognized that sleep has a profound impact on COPD. Sleep played an important role in breathing and gas exchange, poor sleep quality caused an increased risk of aggravation, and sleep-disordered breathing increased the risk of re-hospitalization and mortality [13, 14]. Proper diagnosis and treatment of sleep disorders in COPD were recommended.

Given the high COPD prevalence and burden of COPD patients in China, a better understanding of disease clusters is needed to enable targeted interventions. Therefore, in a relatively large sample of COPD patients (*n* = 223), the objectives of our study were as follows: (1) to identify the symptoms experienced by COPD patients and classify them into symptom clusters based on different symptom dimensions in the stable stage of COPD, (2) to assess the quality of sleep in patients with COPD and compare to symptom and QOL, and (3) to determine the effects of sleep quality and symptom clusters on the QOL of COPD patients.

## 2. Methods

### 2.1. Design and Setting

This survey was conducted between November 2019 and November 2020. 230 patients with COPD were enrolled from the Affiliated People's Hospital of Ningbo University in China. The inclusion criteria of patients were (1) COPD as the primary diagnosis confirmed by respiratory doctors according to Global Initiative for Chronic Obstructive Lung Disease guidelines [15], (2) ≥40 y with stable COPD, (3) no prior history of other major diseases that may affect QOL and symptoms, such as malignant tumor or chronic kidney disease, (4) and agreed to participate in the study. Disease stability was considered to have no exacerbation within 6 weeks prior to study, and all patients were treated for COPD according to the GOLD guidelines (including inhaler evaluation, smoking cessation counseling, and inhaled corticosteroids) [15]. The exclusion criteria were (1) patients with concurrent asthma, bronchiectasis, tuberculosis, or other respiratory diseases and (2) unable to answer the questionnaires. Patients were informed that their participation in the study was voluntary, anonymous, and confidential. Moreover, they had the right to withdraw from this study at any time without any impact on their treatment. Research protocol was approved by the Ethics Committee of the affiliated People's Hospital of Ningbo University (no. 107-W-066).

RETRACTED

### 2.2. Measures

#### 2.2.1. Demographic and Clinical Information

Demographics, including age, gender, marriage, education experience, and professional status, were recorded using general questionnaires. A study-specific questionnaire was developed to gather medical information, including the disease duration, number of exacerbations of COPD in a year, and inhaled drugs therapy. Exacerbations refer to an emergency room visit or hospitalization.

The modified Medical Research Council (mMRC) Dyspnea Scale was used to assess the severity of dyspnea [16], which was one of the most commonly recommended tool. This scale was used widely in clinical trials to estimate respiratory difficulty in COPD patients. This scale was designed with five related questions that were scored from 0–4, and a higher score indicated more severe dyspnea [17].

The COPD Assessment Tool (CAT) was an eight-item, patient-administered questionnaire that was designed for evaluating the severity of disease [18]. The Chinese version of CAT is a reliable, simple, and standardized questionnaire in which patients are required to score eight COPD-related symptoms on a scale from 0 (low impact) to 5 (very high impact), which are then added up to give an overall score of 0 to 40, the higher the score, the more severe the disease status [19]. The CAT is recommended to assess symptoms and patients with a threshold ≥10 which are assigned to the treatment group [20].

#### 2.2.2. Symptom Dimensions

The Revised Memorial Symptom Assessment Scale (RMSAS) [21] was adapted from the MSAS [22], which has been translated into Chinese [23], was used to assess multiple symptoms and to describe multiple aspects of symptoms experienced by patients. Patients were asked whether they had any of these symptoms a week before. If the patients have experienced some of these symptoms, they were then asked to score the frequency, severity, and distress of their symptoms. RMSAS performed well in terms of validity and reliability, and Cronbach's *α* value was 0.86 in COPD patients [21].

RETRACTED

#### 2.2.3. Sleep Quality

In this research, the Chinese version of Pittsburgh Sleep Quality Index (PSQI) was used to evaluate the sleep quality of patients [24, 25]. This tool is a 19-item questionnaire that measures sleep quality for the past month. Each item is rated on a scale of 0–3, and the maximum total score is 21. A total score of PSQI ≥5 indicates poor sleep quality [26].

#### 2.2.4. Quality of Life

The St George Respiratory Questionnaire for COPD (SGRQ-C) was developed to assess QOL in patients with COPD. The scale was adapted and validated from the SGRQ, which was considered to be the gold standard for evaluating QOL in patients with respiratory disease. The SGRQ-C consists of 40 items in three dimensions that are related to symptoms, activities, and effects [27]. Each item is rated from 0 to 100; the lower the score, the better the quality of life [28]. In addition, this tool has been validated in Chinese population [29].

### 2.3. Procedures

The study was conducted in accordance with the Declaration of Helsinki, and all patients had signed the consent forms. Symptoms, sleep quality, and QOL were evaluated by questionnaires at the end of the first month after discharge. The questionnaires were collected by two independent researchers. The demographic information was accessed by patients or their families, and disease information was obtained by researcher from medical records. RMSAS was done independently by the patients. If there were any doubts when filling in the questionnaire, the researcher will be available to help. After completion, the questionnaires were immediately reviewed to make sure that all of the information was obtained.

### 2.4. Statistical Analysis

All analyses were completed with statistical package for the social sciences (SPSS, IBM Inc, Chicago IL; 2011) version 20.0 software. Descriptive statistics were performed for the demographic and clinical characteristics, prevalence, and severity of symptoms. In order to simplify the factor structure, the Kaiser–Meyer–Olkin (KMO) measure and Bartlett's test of sphericity were used in this study. The internal reliability of the symptom clusters was verified by Cronbach's *α*. If the KMO measurement value is ≥0.5 and Bartlett's sphericity test value is <0.05, the data are available for exploratory factor analysis; then, symptom clusters were extracted by performing a principal axis factoring with varimax rotation. The PSQI score ≥5 was used to assign to different sleep quality groups and to compare symptoms and QOL in the groups. Predictors of QOL in COPD patients were analyzed by using binary logistic regression analyses. Variables, such as demographic and clinical characteristics, with possible disparities of QOL, were initially validated by univariate logistic regression. Variables with *P* < 0.1 or variables suspected to be associated with QOL were entered in a binary logistic regression. Cases with missing values were excluded from the analyses. All tests were two tailed, and *P* < 0.05 was considered statistically significant.

RETRACTED

## 3. Results

### 3.1. Demographic Characteristics and Clinical Information

A total of 230 patients with COPD met the eligibility criteria. Seven patients withdrew from our study because they did not return the questionnaires. As a result, 223 patients completed the study. The demographic and clinical characteristics were summarized in Table 1. The mean age of the patients was 65.23 ± 5.64 years, and 68.16% were male. Only 8.52% of the patients had a college degree, 70.8% were married, 82.06% were unemployed, 93.27% of them had no religious beliefs, 87.4% of the patients had smoking history, 69.5% had a disease duration between 2 and 5 years, 68.6% took inhaled drugs therapy, and the mean score of CAT was 20.31 ± 6.47.

### 3.2. Prevalence and Severity of Symptoms

Table 2 includes descriptive statistics of symptom severity and prevalence in the sample. Of all the 19 symptoms, more than 25% of the patients experienced 13 symptoms. The most frequent symptom was cough (*n* = 221; 99.1%), followed by difficulty sleeping (*n* = 210; 94.17%), lack of energy (*n* = 189; 92.2%), shortness of breath (*n* = 188; 91.71%), and feeling nervous (*n* = 172; 83.9%). Symptoms evaluated with the highest severity were as follows: difficulty sleeping, with the median score of 2.98 (1.79–3.58), shortness of breath 2.78 (1.75–3.37), cough 2.53 (1.93–3.14), and lack of energy 2.28 (1.55–2.91).

### 3.3. Symptom Clusters in COPD

Exploratory factor analysis and varimax rotation were performed to extract symptom cluster. Three factors were retained by eigenvalues >1, and three symptom clusters were extracted. Cronbach's *α* of respiratory functional cluster, emotional cluster, and fatigue-sleep cluster was 0.854, 0.841, and 0.847, respectively. The results of factor analysis were summarized in Table 3.

### 3.4. Comparisons of Symptoms and QOL Based on Sleep Quality

To confirm our study hypothesis, we assigned patients into two groups based on the PSQI score of 5. Results of the *t-*test were presented in Table 4. Just as assumed, the poor sleep group was obviously different from the normal sleep group on the SGRQ-C, except for the SGRQ symptom score. The RMSAS revealed a significant difference between the two groups, except for worrying in cluster two.

RETRACTED

### 3.5. Factors Affecting QOL

Logistic regression analyses were used to identify factors influencing QOL, and the results were shown in Table 5. The following are the demographic and clinical characteristics with statistical differences, age, education status, marital status, work status, medical insurance, and disease duration as verified by univariate analysis, were put in as independent variables. Three symptom clusters and PSQI scores were also put in as clinical study variables. The results revealed that QOL in COPD patients were most influenced by sleep quality and respiratory functional cluster.

## 4. Discussion

This study evaluated clinical symptoms, sleep quality, and QOL in COPD patients. The symptoms of COPD patients were studied and separated into three symptom clusters. Sleep quality and QOL were also assessed then to identify factors affecting QOL in patients with COPD. Our study suggests that appropriate interventions based on symptom cluster may be effective in improving symptom management and QOL in these patients.

In this study, symptoms experienced among COPD patients were described by using RMSAS. The common symptoms in this study were cough, sleep disorder, and shortness of breath, which were similar to previous studies [30, 31]. However, COPD patients in our study were more likely to report anxiety, feeling nervous, sad, and irritable. Unlike previous studies, there were fewer symptoms of numbness or tingling in hands/feet [31]. This result indicates that the mental state should be paid more attention and managed. In terms of severity, sleep disorder had the highest level of severity, which was inconsistent with previous studies [30, 31]; the difference may be owing to all the involved participants in previous studies with severe or acute COPD, whereas most of our participants had stable COPD. Therefore, health staff should be concerned about the sleep quality of COPD patients after discharged from hospital.

The 13 symptoms described in our study were categorized into three symptom clusters. Factor 1 included five symptoms: shortness of breath, dry mouth, cough, feeling bloated, and problems with sexual interest or activity. Yang et al. examined 19 symptoms of patients with exacerbation of COPD and identified shortness of breath, cough, dry mouth, feeling drowsy, and fatigue, as a symptom cluster [32]. In South Korea, patients with COPD were from a university hospital; their symptoms were classified into dyspnea, dry mouth, and physical functional status, as a single symptom cluster [33]. As demonstrated above, COPD patients exhibit similar symptoms related to respiratory function.

RETRACTED

Factor 2 consisted of feeling nervous, feeling irritable, worrying, and I do not like myself. Kyeung et al. considered anxiety and depression as a single symptom cluster in COPD patients, named the mood cluster [33]. Feeling drowsy, feeling nervous, feeling sad, feeling irritable, and worrying are characteristic symptoms of AECOPD, so factor 2 in this study was named the emotional cluster [32]. These results were similar to the findings of our study. Patients with COPD are reported to be anxious for fear of recurring shortness of breath after their first appearance [33]. The results of this study suggest that health care providers should strive to understand patients, assess their psychological symptoms, and take appropriate intervention measures.

For factor 3, this symptom cluster included three symptoms: lack of energy, feeling drowsy, and difficulty sleeping. Sleep disturbances are linked to several respiratory diseases, including COPD. Decreased sleep quality is always described in COPD patients, which is likely to play an important role in chronic fatigue and decreased quality of life [34, 35]. In one study, sleep disorder and fatigue constituted a symptom cluster that was consistent with the results of our study. Thus, factor 3 in our study was labelled as fatigue-sleep cluster. In addition, attention should be paid to the sleep disturbance in COPD patients, which represents underexplored way to improve QOL among these patients.

In this study, sleep quality of COPD patients was measured by the PSQI; 70.4% of the patients valued above 5 points, which indicated as poor sleep quality in this scale. This percentage is lower than that for COPD patients in Turkey, which is 94% as measured by using the same instrument [36]. Moreover, PSQI was negatively correlated with QOL, with most COPD patients having poor sleep quality. This indicates that health professionals should be aware of sleep disorders in COPD patients and provide appropriate interventions to improve sleep.

This study indicates that factors affecting the QOL of patients are sleep quality and the respiratory functional cluster. Respiratory functional cluster was shown to affect the QOL, suggested the importance of active treatment and interventions.

Finally, sleep quality was identified as an important factor influencing patients' QOL. Poor sleep quality can lead to exacerbation and mortality [36]. Factors that contribute to sleep disorder in COPD patients have been described as cough, dyspnea, and sleep apnea. There were few studies reported in the relationship between sleep quality and QOL in patients with COPD. Buket et al. investigated the relationship between sleep quality and QOL in patients with moderate to severe COPD and found that PSQI was negatively correlated with QOL [37]. Although 157 patients (70.4%) of this study were considered to have poor sleep quality, only 19 patients (12.1%) were taking medicine to improve sleep quality. This means that only a low proportion of COPD patients with sleep disorders actually receive interventions to improve their sleep. Although there are various reasons for the discontinuity between the sleep assessment and therapeutic interventions, the main reason is lack of sleep health service and lack of awareness among health staff.

RETRACTED

This study has some limitations. Firstly, all of the participants were stable COPD patients at a single center, which limits the generalizability of the study's conclusions. Secondly, this study was a descriptive study design and could not determine longitudinal changes in symptom clusters associated with COPD. Finally, we cannot determine the causality because of the complex interplay among sleep quality, symptom clusters, and QOL.

## 5. Conclusion

This study explored the symptoms of patients with COPD and divided them into three symptom clusters. The three symptom clusters will be benefit for managing symptoms of COPD patients. Sleep quality and QOL among COPD patients were also examined to identify the factors affecting their QOL. The respiratory functional cluster and sleep quality were confirmed as risk factors affecting the QOL in our study and should be used as the basis for developing intervention programs to improve the QOL of patients with COPD.

## Figures and Tables

**Table 1:** Demographic and clinical characteristics of the participants (*n* = 223).

Characteristic	*n* (%) or mean (SD)
*Demographic characteristics*	
** **Age, y	65.23 (5.64)

** **Gender	
** **Male	152 (68.16)
** **Female	71 (31.84)

** **BMI (kg/m^2^)	
** **≤18.4	53 (23.77)
** **18.5∼23.9	112 (50.22)
** **24∼27.9	42 (18.83)
** **≥28	16 (7.18)

** **Educational level	
** **High-school degree or less	201 (90.13)
** **College graduate	22 (8.52)

** **Marital status	
** **Married	163 (70.8)
** **Divorced or separated	60 (26.9)

** **Work status	
** **Employed	40 (17.94)
** **Unemployed	183 (82.06)

** **Religious belief	
** **Buddhism	9 (4.03)
** **Christianity	3 (1.35)
** **None	208 (93.27)

** **Medical insurance	
** **Yes	219 (98.2)
** **No	4 (1.79)

** **Monthly income, RMB	
** **<2000	19 (8.52)
** **2000∼4999	163 (73.09)
** **≥5000	41 (18.3)

** **Smoking status	
** **Former or current	195 (87.4)
** **Never	28 (12.56)

*Clinical characteristics*	
** **Disease duration, y	
** **<1	29 (13.0)
** **2∼5	155 (69.5)
** **>5	39 (17.5)

** **Inhaled drugs' therapy	
** **Yes	153 (68.6)
** **No	70 (31.4)

** **Number of exacerbations of COPD, per year	
** **0	44 (19.73)
** **1∼5	160 (71.75)
** **≥6	19 (8.52)
** **CAT	20.31 (6.47)

** **mMRC grade	
** **0	3 (1.34)
** **1	53 (23.8)
** **2	62 (27.8)
** **3	92 (41.3)
** **4	13 (5.83)

Notes: BMI, body mass index; RMB, Ren Min Bi; inhaled drugs' therapy, treatment with inhaled corticosteroid; mMRC, modified Medical Research Council Dyspnea Scale.

RETRACTED

**Table 2:** Prevalence and severity of 19 symptoms in participants (*n* = 223).

Symptoms^a^	Occurrence	Severity^b^
	*n* (%)	Median (interquartile range)
Shortness of breath	188 (91.71)	2.78 (1.75–3.37)
Dry mouth	105 (51.22)	1.54 (0.97–2.54)
Lack of energy	189 (92.2)	2.28 (1.55–2.91)
Cough	221 (99.1)	2.53 (1.93–3.14)
Feeling nervous	172 (83.9)	2.05 (1.33–2.61)
Feeling sad	155 (75.61)	1.62 (1.01–2.27)
Feeling irritable	162 (72.65)	1.44 (0.80–2.01)
Worrying	168 (79.02)	1.56 (1.03–2.42)
Feeling drowsy	164 (80)	1.13 (0.57–1.65)
Difficulty sleeping	210 (94.17)	2.98 (1.79–3.58)
Feeling bloated	112 (54.63)	0.55 (0.00–0.97)
Pain	57 (21.8)	0.23 (0.00–0.83)
Numbness or tingling in hands and/or feet	47 (22.93)	0.25 (0.00–0.99)
Difficulty concentrating	41 (20)	0.19 (0.00–0.56)
Sweats	25 (12.2)	0.12 (0.00–0.45)
Problems with sexual interest or activity	108 (52.68)	0.47 (0.00–0.78)
Swelling of arms and/or legs	55 (24.83)	0.38 (0.00–1.03)
I do not look like myself	169 (82.44)	1.24 (0.65–1.77)
Changes in skin	47 (22.93)	0.19 (0.00–0.61)

Notes. ^a^Symptoms from the Recised Memorial Symptom Assessment Scale. ^b^Severity: 1, slight; 2, moderate; 3, severe; 4, very severe.

**Table 3:** Exploratory factor analysis using ratings of symptom severity (*n* = 223).

Symptoms	Factor 1	Factor 2	Factor 3
	Respiratory functional cluster	Emotional cluster	Fatigue-sleep cluster
Shortness of breath	0.712		
Dry mouth	0.643		
Cough	0.799		
Feeling bloated	0.637		
Problems with sexual interest or activity	0.615		
Feeling nervous		0.694	
Feeling sad		0.701	
Feeling irritable		0.687	
Worrying		0.753	
I do not look like myself		0.644	
Lack of energy			0.733
Feeling drowsy			0.684
Difficulty sleeping			0.772
Cronbach's *α* coefficients	0.854	0.841	0.847
Eigenvalue	3.31	3.54	2.87
Explained variance	2.01	2.17	1.85
Explained (%)	43.73	47.28	39.64
Cumulative (%)	28.82	21.40	39.60
Kaiser–Meyer–Olkin		0.885	
Bartlett sphericity test		<0.001	

**Table 4:** Quality of life, symptom scores, and sleep quality in poor sleep and normal sleep groups determined by the PSQI.

Variable	Total (*n* = 223)	Poor sleep group (*n* = 157)	Normal sleep group (*n* = 66)	*P*
**QOL**				
** **SGRQ symptom score	54.7 (20.4)	55.1 (22.3)	51.3 (19.1)	0.082
** **SGRQ activity score	64.7 (29.5)	70.2 (20.8)	61 (33.8)	**0.015**
** **SGRQ impact score	39.1 (21.3)	46.9 (18.1)	31.1 (16.4)	**0.004**
** **SGRQ total score	52.3 (22.1)	57.1 (19.3)	47.4 (27.9)	**0.006**

**Symptom cluster**				
** **Factor 2				
** **Feeling sad	1.62 (1.01–2.27)	2.45 (1.42–3.01)	1.13 (0.57–1.65)	**<0.0001**
** **Feeling irritable	1.44 (0.80–2.01)	2.23 (1.27–2.87)	0.92 (0.45–1.33)	**<0.0001**
** **Worrying	1.56 (1.03–2.42)	1.64 (1.03–2.29)	1.09 (0.51–1.87)	0.058
** **Factor 3				
** **Lack of energy	2.28 (1.55–2.91)	3.04 (1.87–3.36)	1.55 (1.01–2.38)	**<0.0001**
** **Feeling drowsy	1.13 (0.57–1.65)	2.15 (1.13–2.67)	1.02 (0.47–1.65)	**0.001**
** **Difficulty sleeping	2.98 (1.79–3.58)	3.31 (2.11–3.67)	2.14 (1.28–2.98)	**<0.0001**

RETRACTED

**Table 5:** Logistic regression analysis model of quality of life (*n* = 223).

Variable	*B*	SE	Wald *X*^2^	*P*	OR	95% CI
Age	0.045	0.027	3.165	0.085	1.056	0.975–1.189
Disease duration, y						
** **<1	0.456	0.876	0.285	0.591	1.583	0.312–8.753
** **2∼5	0.322	0.492	0.433	0.509	1.387	0.534–3.700
** **>5	0.857	0.612	2.115	0.153	2.575	0.758–7.981
PSQI	−1.927	0.687	7.628	**0.007**	0.158	0.038–0.579
Factor 1	−0.803	0.075	3.547	**0.001**	0.467	0.101–1.023

## Data Availability

All data supporting this study is provided as supplementary information accompanying this paper. The data used to support the findings of this study have been deposited in the (Effects of Symptom Clusters and Sleep on the Quality of Life in Patients with Chronic Obstructive Pulmonary Disease) repository (DOI Number https://doi.org/10.1155/2021/1692480). The investigation data used to support the findings of this study were supplied by Shanghai Jiaotong University, School of Medicine under license and so cannot be made freely available. Requests for access to these data should be made to the corresponding author. The investigation data used to support the findings of this study are restricted by the Ethics Committee of the affiliated People's Hospital of Ningbo University in order to protect patient privacy. Data are available from the corresponding author for researchers who meet the criteria for access to confidential data. The investigation data used to support the findings of this study are available from the corresponding author upon request.
